The article "Detection of Fake News Text Classification on COVID-19 Using Deep Learning Approaches" was published in 2021. Journal: Comput Math Methods Med.

# Detection of Fake News Text Classification on COVID-19 Using Deep Learning Approaches

**DOI:** 10.1155/2021/5514220

**Published:** 2021-11-15

**Authors:** Waqas Haider Bangyal, Rukhma Qasim, Najeeb ur Rehman, Zeeshan Ahmad, Hafsa Dar, Laiqa Rukhsar, Zahra Aman, Jamil Ahmad

**Affiliations:** ^1^Department of Computer Science, University of Gujrat, Pakistan; ^2^Department of Software Engineering, University of Gujrat, Pakistan; ^3^Professor Computer Science, Hazara University, Manshera, KPK, Pakistan

## Abstract

A vast amount of data is generated every second for microblogs, content sharing via social media sites, and social networking. Twitter is an essential popular microblog where people voice their opinions about daily issues. Recently, analyzing these opinions is the primary concern of Sentiment analysis or opinion mining. Efficiently capturing, gathering, and analyzing sentiments have been challenging for researchers. To deal with these challenges, in this research work, we propose a highly accurate approach for SA of fake news on COVID-19. The fake news dataset contains fake news on COVID-19; we started by data preprocessing (replace the missing value, noise removal, tokenization, and stemming). We applied a semantic model with term frequency and inverse document frequency weighting for data representation. In the measuring and evaluation step, we applied eight machine-learning algorithms such as Naive Bayesian, Adaboost, *K*-nearest neighbors, random forest, logistic regression, decision tree, neural networks, and support vector machine and four deep learning CNN, LSTM, RNN, and GRU. Afterward, based on the results, we boiled a highly efficient prediction model with python, and we trained and evaluated the classification model according to the performance measures (confusion matrix, classification rate, true positives rate...), then tested the model on a set of unclassified fake news on COVID-19, to predict the sentiment class of each fake news on COVID-19. Obtained results demonstrate a high accuracy compared to the other models. Finally, a set of recommendations is provided with future directions for this research to help researchers select an efficient sentiment analysis model on Twitter data.

## 1. Introduction

NLP a specified area of research which deals with the phenomena how computers can take part in understanding and manipulating human language (text and speech) to perform useful operations. It is an area in which after analyzing the data, proposed model can grab relevant or useful data using context and input can be represented in a different way [1]. In recent decades, artificial intelligence (AI) has changed our lives and developed rapidly in no time. NLP is AI technology that is involved in text classification, information storage and retrieval, information extraction, semantic analysis, machine translation, dialogue system, speech recognition, and much more [2]. AI technology is very popular for smart homes, smart industries, smart transportation, smart healthcare, smart cities, and satellite. It comprises many IoT devices (Things) that are equipped with different sensors, actuators, storage, computational, and communicational capabilities to collect and exchange the data over traditional internet. The data that is being captured and processed within the IoT network is of sensitive nature that demands security from possible intrusions. Different security mechanisms such as firewalls, authentication schemes, different encryption methods, and antiviruses are currently used to protect sensitive data from possible security attacks. Natural language processing allows the system to perform operations on natural human language and translates it to machine understandable format [3]. [4] states in their research that practical swarm optimization (PSO) algorithm is a complex method of searching used for food in a different manner of bee swarming. Multiple problems of optimization are solved using PSO. They proposed a technique termed as WE-PSO, which incredibly solves the optimization issues. They had evaluated their proposed model on fifteen different well know tasks. Results had showed that WE-PSO performs this task incredibly well as compare to other multimodal and unimodal techniques. Metaheuristic algorithm is used for text and data classification tasks [5–9]. These algorithms provide better performance in feature extraction phase of text phase as well [10–15].

Due to big data generated by users on social media, the amount to hate speeches is also increased. Natural language processing is focusing on hate speech detection on social media and particularly the automatization of this task to detect hatred speeches on social platforms [16]. (Mustafa et al., 2017) used Urdu fake news on COVID-19 to detect the controversial Urdu speeches on twitter. Natural language processing can also be used to explore his effect on social justice with society. NLP techniques can be used to detect fake reviews [17]. [18] provides a comprehensive overview in his work that how natural language processing is applicable in psychology. [19] provides a comprehensive literature review of NLP and text mining in bioinformatic field. [20] describes in their research that artificial neural network is used in many classification tasks, but this traditional technique has some drawbacks. To overcome these drawbacks, they had trained a neural network opposition based practical swarm optimization. They had also performed a performance analysis which showed that (OPSONN) performs efficiently best among other methods.

User generated content (UGC) on different social interaction handles is a new source of data for scientist and industry. UGC on review sites contains important information in textual form and has to extract using SA and opinion mining techniques [21]. One of the important aspects of personal growth and development is understanding human emotion. Emotions and behaviors hold massive importance in human-human effective and successful communication. Sentiment analysis and affective computing have the ability to enhance the capabilities of the recommendation system and customer relationship management [22]. Work done by [23] describes an NLP-based approach to process customer generated content (hotel reviews) and produce valuable insights form it. [24] had developed a prediction model for online hotel reviews to predict the helpfulness of reviews. Sentiment analysis is the study of opinions which are expressed in piece of text written by user/customer. This opinion describes the positive, negative, or neutral behavior/attitude of user/customer. This research mainly focuses on implementation of different machine learning classification algorithms for analyzing the restaurant reviews. And SVM performed better for given dataset [25, 26]. A forward only counter propagation network-based approach used to diagnose the contraceptive method choice disease. Their research work proposes a method named as forward only counter propagation network (FOCPN) for resolving classification tasks for medical field. Performed experimentation and results clearly show that proposed model convergence is really fast, and the efficiency and reliability have higher scores.

Word embedding is one of the useful and significant approaches for several natural language tasks. In this research, they proposed an approach that uses sentiment prior knowledge from both levels: document and word level [27]. Research done by [28] presented their method for twitter data SA which uses word embedding method considering co-occurrence statistical characteristics and latent contextual semantic relationships. [29] proposed a fuzzy approach for SA, using fuzzy membership degrees. They compare the performance of their approach with mostly used sentiment classifiers, and results showed that their approach performs marginally better. A topic base sentiment analysis approach was proposed by [30] for understanding the user opinion in Twitter. The research mainly focuses to identify cultural, economic, environmental, and social factors related to public health and environment. They had used the #WordEnviromentDay to generate dataset. Bat algorithm is a type of algorithm which is inspired by nature. It is used to solve the problems of optimization. BA has some limitations, and this research work proposes a news aspect of BA and named it as IBA. This variant modifies and enhances the abilities of local minima. Results show that proposed method outperforms than traditional neural network.

Sentiment mining is the type of textual data analysis which filter the words and sentences with high frequency and hold meaningful information. As sentiment refers to feelings or attitudes, so we can say that, sentiment analysis is used to obtain, highlight and analyze hidden sentiments. With the rapid generation of big data from Internet and online communities, this data can be utilized for investment decision making. For this purpose, [31] proposed a dynamic prediction approach for online financial communities behavior, stock market, and perspectives of behavioral finance using news articles and blogs related to finance [32]. Microblogs are the common platforms for users to discuss about society, environment, technology, science, entertainment and so on. This data reflects the user point of view about a topic which can be negative, positive, or neutral. They proposed an approach to classify the text on Chinese microblogs about a topic that is positive, negative, or neutral. Sentiment mining or sentiment classification is a very difficult and sensitive task of mining important and useful information from text available on online social media sites.

In past years, an interesting area of research is solving the problems of stock forecasting with time series. Work done by [33] proposed an approach which uses financial microblogs for stock market forecasting considering time series of stock index and time series of sentiment. [34] states in their research that many techniques for topical detection and sentiment detection consider important microblogging data as noise. To solve this problem, they had presented a multimodal which is further joined with sentiment topic model for SA of microblogs. [35] elaborates the concepts of concept-level analysis of sentiments. It uses the concepts and characteristics of reviews which are provided by users. Earlier studies used bounded pair of rules for concept level sentiment classification. So, this research proposed a set of rules to overcome these limitations of concept level sentiment analysis. Proposed system appears very effective with 87.5% of accuracy score.

The rest of the paper is organized as follows: Section 2 discusses literature review.  Section 3 discusses the types of classification algorithm.  Section 4 overviews methodology. Experimental results are discussed in Section 5. The conclusion and future prospects of our work are discussed in Section 6.

## 2. Literature Review

According to [36], traditional natural language processing techniques are not that much feasible to be applied on big data for detecting sentiments. Therefore, they proposed a model by integrating self-organization map, principle component analysis, and Adam DL for unsupervised machine learning, dimensionality reduction, and computational classification, respectively. Further, they performed a comparative study between proposed approach and state of art approaches. They used seven datasets containing 15 k, 30 k, 45 k, 60 k, 75 k, 90 k, and 100 k, respectively. Classification accuracy of all datasets is 84.67%, 85.12%, 85.89%, 86.78%, 87.21%, 87.63%, and 88.34%, respectively. Result shows an interesting phenomenon that by using a bigger size of data performance of presented model also increased. They studied four algorithms (PCA-based CNN, LR, polynomial regression, and RF) in their research and conclude that proposed approach has high accuracy 88.34% among all.

[37] states in their research that most studies on aspect-level categorization of sentiments are based on supervised machine learning which definitely needs labeled sample data. To solve this issue, they presented an aspect level sentiment categorization with semisupervision based on variational autoencoder (AL-SSVAE). Proposed model inputs a given aspect as encoder and decoder based on VAE (variational autoencoder) and then added a classifier which is ATAE-LSTM. They compared their model with LSTM, AE-LSTM, AT-LSTM, and ATAE-LSTM to show that their model performs better. Results clearly show that AL-SSVAE leads among all models on all four datasets. Accuracy percentages of proposed model on all datasets CAME, PHNS, REST, and LAPT are 79.72%, 80.66%, 86.72%, and 88.98%, respectively

[38] states in their research that CNN has gained promising focus and discussion in the area of sentiment classification. They also used CNN for classification of data on the bases of sentiments but add consecutive convolutional layers for this purpose and also compare this model with other state of the art deep learning approaches as well as with machine learning approaches using three different datasets. Their proposed CNN model contains an embedding layer, two convolutional layers, a pooling layer, and a fully connected layer. Many machine learning studies focus on two or more than two sentiment labels. Proposed CNN model is compared with NB, DT, SVM, and RF. Results clearly show that consecutive layer CNN is leading with 81.06%, 78.3%, and 68.3% accuracy using movie review, customer review, and Stanford sentiment treebank datasets, respectively. They had also tested their model on ternary classification and applied the model on MR Dataset. Their model leads with 68.3% accuracy among all ML and DL models

Work done by [39] describes in their research, and emotions shared on social networking sites can be utilized by many useful purposes. They have done sentiment analysis on movies dataset IMDb using a hybrid feature extraction model. They joined the TF and TF-IDF machine learning features along with lexicon features. They have compared the machine learning models with their hybrid model which leads in terms of complexity and accuracy. After experiment, results clearly show that when different machine learning classifiers like SVM, NB, KNN, and maximum entropy are used with feature selection method along with hybrid features, it gives promising results in terms of accuracy and complexity.

[40] describes in their research most of the literature on sentiment classification used approaches based on lexicon or ML techniques. Previous researches also only consider binary classification while ignoring neutral review. Drawback of lexicon approach and ML approach is the system depends on lexicon dictionary and resource and system's performance depends upon algorithms, respectively. To solve this problem, the proposed a hybrid model which uses combination of machine learning algorithm (SVM, NB, LR, and DT) and lexical approach (SentiWordNet). Three different datasets IMDB, Amazon product review dataset, and Twitter dataset are used for classification and sentiment analysis purpose. Performance of four machine learning classifiers is tested with and without using lexicon approach. Results demonstrate that all classifiers perform better with lexicon approach in the context of perception, recall, and accuracy, but SVM and LR outperform among all.

[41] states in their work that correctness of sentimental analysis work relies on domain specific dictionary completely based on correctness of that dictionary. To solve this issue, they proposed a method which uses emotional characteristics from review's fragment instead of whole review with conditional random field algorithm (CRF). Then, they assign weights to feature words asymmetrically and apply SVM for classification purpose. They gathered data from two resources. One dataset is gathered from Chinese review site about Audi A4 car, and other dataset is collected from Amazon website about Samsung S7 phone. They performed three different experiments and used (CRF+ asymmetric weighting+ SVM), (TDIDF+SVM) ,and (CRF + TDIDF+SVM), respectively, on 1, 2, and 3 using these two datasets. After experiments were performed, results clearly show that average accuracy of Chinese dataset increased to 90%, and average accuracy of English dataset also increased to 91% using conditional random field algorithm and asymmetric weighting.

[42] describes in their contributed work that many research work on sentiment analysis through machine learning uses text, emoticons, or images solely. Text with combination of emoticons has always been neglected. So, they proposed a model and algorithm to find SA using text and emoticons both. They analyzed both text and text with emoticons using ML and DL separately and also combined. They collected data from Twitter about Airline reviews. They also generated the emoticons, and lexicon contains vastly used emoticons by all users on Twitter and used it in their research. They used SVM, NB, LR, Random Forest, LSTM, and CNN for analysis of machine learning and deep learning algorithm. LSTM and CNN outperforms among all algorithms with accuracy of 0.89, 0.81, 0.88, and 0.79 on (text+ emoticons) and text, respectively. This clearly shows that deep learning algorithms perform better than machine learning algorithms. They also compared their proposed model with existing models, accuracy of text SA increases from 57 to 78, and accuracy of text and emoticons raised from 65 to 89 with proposed model.

[43] performed SA study on drug reviews. They state in their research that medical and health reviews are not much analyzed by researches of NLP and DM. They proposed two fusion models named as 3W1DT and 3W3DT. First fusion model has combination of deep model with a traditional learning algorithm (GRU, CNN, and 3CRNN with NB, DT, RF, and KNN). And second fusion model has three deep models with one traditional model. They used drug review dataset containing 215063 reviews in total categories as positive, negative, and neutral. When the experiments are performed on dataset, after first experiment between seven different algorithms NB performs good among all. When second experiment with 3W1DT was performed, 3CRNN-NB performs good among all. When third experiment was performed using 3W3DT, NB outperforms with second fusion model with high accuracy among all. After that, they compared their best model 3W3DT-NB with already existing model, and proposed model leads with accuracy of 88.36%

[44] presented general machine learning method with *n*-gram IDF feature extraction. After feature extraction, an automated ML tool was used for distribution of data according to sentiments. They used a dataset that contains documents related to mobile application review, question answers related to stack overflow, and different comments on Jira issue. They distributed their datasets into positive, neutral, and negative subdocuments as per their method requirement. Firstly, they apply text processing on their datasets. After that, they used *n*-gram IDF for feature extraction. Then, they used sklearn for automatically classifying reviews or comments into positive, negative, and neutral. Results clearly show that their presented model outperforms among all existing models with high accuracy of correct predictions. In stack overflow, app review and Jira issue accuracy rate was 1317/1500, 293/341, and 884/926.

[45] states in their research that twitter data on politics holds great importance for political parties, as they can predict sentiments of their supporters from their tweets. They proposed a model which uses two *n*-gram hybrid technique and NB for classification purposes. This model improves the precision and recall accuracy of *n*-gram models by solving “zero count problem.” Proposed approach performs sentiment analysis in two phases and applies two *n*-gram models: least-order *n*-gram model and highest-order *n*-gram model. They used OMD (Obama McCain) dataset as benchmark. After the experiments were performed, proposed algorithm performs well among all previous studies that were performed on same dataset. This model increases accuracy of unigram model to 76.14%, *n*-gram model to 67.00%, and hybridized model to 80.00%. It shows that using both unigram and *n*-gram model combined can predict the sentiments more accurately.

[46] worked on targeted sentiment analysis which focuses on detecting sentiments on a particular topic. They mentioned that most of previous researches used RNN with context and target words to detect target sentiments. To overcome this issue, this study presented a model named as attentional encoder network. This model keeps RNN away and uses attention instead, and model uses layers like embedding layer, attentional encoder layer, target specific layer, and finally the output layer. Here, embedding layer is further divided into two types named as AEN-GloVe and AEN-BERT. They used three datasets for evaluation purposes. SemEval 2014 task 4 contains restaurant reviews and laptop reviews. Other dataset named as ACL 14 contains Twitter data. These datasets further divided as positive, neutral, and negative. Results clearly show that their proposed models AEN-GloVe, AEN-BERT, and BERT-SPC perform better among all analyzed approaches.

[47] states in their research that aspect-level analysis holds great importance but the main hurdle in this research area is labeled data relative to aspect-level analysis. So, they proposed a model called transfer capsule network (TransCap). This basically transfers document level knowledge to aspect level knowledge. They evaluate their approach using two datasets of restaurant and laptop reviews obtained from SemEval 2014 task 4. For knowledge transfer purpose of documents, they used Yelp, Amazon, and Twitter reviews. After evaluation, results clearly show that proposed approach reaches to 79.5% and 73.87% accuracy on restaurant and laptop dataset, respectively, among all analyzed techniques.

[48] describes in their research work that DL approaches are used vastly for opinion mining, sentiment mining, document classification, document clustering, etc. They performed comprehensive study on DL models for SA. CNN and LSTM are of main concern. They analyzed all previous techniques on Turkish movie reviews obtained from a Turkish website. They checked the effect of word embedding with these techniques and also developed some variants of CNN and LSTM models by changing the layers in it. After the experiments, results clearly showed that using PWE (pretrained word embedding) with all deep learning models improves their accuracy. The highest test accuracy 98% was achieved by CNNLSTM.

[49] evaluated DL models for fake news detection using Contraint@AAAI 2021 COVID-19 fake news detection dataset. Used classification algorithms rely on CNN, LSTM, bi-LSTM+attention, HAN (hierarchal attention network) BERT-base, and DistilBERT. Their aim is to classify the news as fake or real. This task is also considered as classification task of text. They were mainly focused on what was written in news, and they completely forget other features like user characteristics and social circle. BERT and DistilBERT approaches which are pretrained on the COVID-19 tweet corpus showed the best performance among all other which only finetuned on the dataset. Model named as BERT-cased which was trained manually on the COVID-19 tweet corpus and joined with Covid-Twitter-BERT approach performs better. HAN performed the best as compare to all nontransformer approaches

[50] performed a sentence-level classification task. They performed multiple tests with CNN trained on top of pretrained word vectors for sentence-level classification tasks. They try CNN in combinations with (Word2Vec + CNN, GloVe+CNN, ELMo+CNN and BERT+CNN). Results clearly showed that BERT+CNN performs better than all other combinations on two datasets, respectively: manifestos project corpus for training the model and coronavirus (COVID-19) press briefing corpus for testing the performance of model. BERT+CNN achieves 68.65% accuracy and 64.58% F1 score.

[51] states in his research that supervision of human and detection of wrong stories is nearly impossible task. With advancement in processing techniques, ML models, DL models, and user involvement can be replaced by assigning pattern identification task to computers, but it requires a large dataset of both real and fake news. He collected the news around the word from 15 January 2020 to 15 February 2020 but the data was unlabeled. After removing unnecessary data and labeling the news articles, dataset contains 2426 articles labeled true and 1646 articles labeled false. After classification experiments, LR achieved 75.65% accuracy, embedding with dense layer achieved 86.93% accuracy, embedding with LSTM layer achieved 86.9% accuracy, and bi-LSTM model achieved 72.31% accuracy.

[52] states in their research that fake news have important role in everyone's life in these days. An individual's life can totally change due to these fake COVID-19 news. The authors introduced a method to check the sentiments of real and fake news based on COVID data. They performed text classification with the model based on additional neural classification head built with multiple hidden layers. Dataset consist of COVID-19 content in English from Twitter, Facebook, and Instagram. They split the dataset into three parts: train, validation, and test. The proposed model outperforms among all uses stacking, where they combine different neural and nonneural features sets. This models achieves the 0.972 F1-score.

[53] introduced a technique to detect the misleading information about corona-virus. Their trained model relay on the shared data about COVID-19 on different platforms using different accounts like WHO, UNICEF, UN, and from reliable websites. They have built an ensemble system that used multiple DL techniques to detect misleading information. They have also used two steps to improve the performance of their system: data preparation and data preprocessing in combination with feature engineering step. They examined their model's performance using fourteen different parameters. Results are promising and contain high accuracy. [54] states in their research that there is bulk of misleading COVID-19 data on social media. Their research proposed an application (CO-verified) that uses machine learning and human power as well to access the credibility of news. They also train bi-LSTM model on 1275 news pieces from GoAID and achieve 0.93 F1 score.

[55] elaborated the impact of social media in our daily lives. They also highlighted the misleading information on social media and its effect on our lives. They proposed an approach to detect the fake and real news about coronavirus. Model achieves high F1 score and occupied second position on leaderboard. They used the dataset generated by (patwa et al., 2020) containing posts and tweets collected from Facebook, Twitter, and Instagram. They have split the dataset into train test and validation parts. They tried different baseline models on this dataset like NB, SVM, LR, and XGBoost. They have also use different transformers models. Their electra model achieves the 0.9827 F1-score on official test set.

[56] says in their research that fake news related to coronavirus are spreading faster than the real facts. And these fake tweets are putting people's lives on high risk. They introduced first coron virus twitter dataset called CTF and also, they contributed more through proposing a model for detecting real and fake tweets called cross-SEAN (crossstitch-based semisupervised end-to-end neural attention model). CTF dataset contains 45.26 k tweets in total in which 18.55 k are labeled as genuine and 26.71 k are labeled as fake. They compared the behavior of their model with seven existing approaches, and their model outperforms all by achieving the 0.95 F1 score [57]. Fake news has gain immense popularity for social, business, and political reasons. News related to coronavirus has left great impact on offline community as well. In these situations, it becomes more important to distinguish between real and fake COVID-19 news to avoid the fear of this dangerous virus. They used the dataset generated from web concerned with binary classification of COVID-19 fake news. They applied preprocessing to dataset and use TF and IDF for feature extraction. After that, they train their model using decision tree and random forest and evaluate their model using different parameters. Proposed model achieved 94.49% accuracy with RF classifier and 92.07% accuracy with DT.

[58] applied classical ML algorithms combined with multiple linguistic features including reliability, *n*-gram, punctuation, and emotional tone. His research uses different experimental preprocessing steps. Performance of system is measured using F1-score parameter along with accuracy, recall, and precision. Experiments are performed with different preprocessing and features sets. NB, RF, SVM, LR, and multilayer perceptron are used. Model which achieves the highest performance is based on linear SVM with 95.70% F1-score beating baseline model for this dataset. And the second best performing model was logistic regression with 95.42% F1-score.

## 3. Types of Classification Algorithm

There are many classification algorithms available in machine learning and deep learning which can be made available in various instances. The major classification algorithms are listed below:

### 3.1. Support Vector Machine (SVM)

SVM is an ML classifier that we have applied in our study. SVM applies to both linear and nonlinear problems and has given significant results for many real-life applications [59]. SVM separates the data into classes with the help of a line/hyperplane. It works best for non-inear problems due to its functions known as kernels that take input space in low dimensions and convert it into high dimensional space. Shortly, SVM is capable of performing highly complex data transformations and separating data into respective classes.

### 3.2. Logistic Regression (LR)

LR is one of the most widely used classification algorithms. It is a statistically based model that makes use of a vector of variables and finds out the weight for each variable and based on this predicts the class of stated fake news on COVID-19 in the form of word vector. LR can only be used when the dependent variable is dichotomous (binary). In LR, there is no linear relationship between the dependent and independent variable, and the independent variable neither be normally distributed nor of equal variance within a group [60].

### 3.3. Naïve Bayes

NB is a probabilistic classifier that is based upon Bayes theorem. The main reason for its popularity is its simplicity, accuracy, and reliability. It has been applied to various real-life applications, but it has found most applications in natural language processing problems. The basic assumption of NB is each feature makes an equal and independent contribution in the outcome, and this is why NB is called “Naive.” It calculates the probability of an attribute using preceding information that may be related to that attribute.

### 3.4. Adaboost

Adaboost also known as adaptive boosting is the very first boosting algorithm in machine learning. Boosting algorithms are well known for converting lazy learners into eager learners [61]. It is mainly used to improve the prediction capability of lazy learners by training them. Adaboost combines multiple slow learners and makes one strong learner from them. It works iteratively. Initially, all the instances are assigned similar weights and in the next iterations, weights of wrongly categorized instances are updated; as a result, the weights of correctly classified instances decrease, and the weights of misclassified instances increase.

### 3.5. *K*-NN

KNN is a classification algorithm that classifies the instances to the nearest neighbor with the majority vote. To find the nearest neighbor, the classifier uses the distance metric and finds out the neighbor with the smallest distance. The distance is taken between the test instances and all the training instances. The distance can be measured using known distance measures such as Euclidean distance [62]. A specific value is gained using all nearest neighbor training examples and then takes that number which one appears most as prediction value and categorizes the new test dataset. KNN gives highly accurate predictions; therefore, it is used for applications that require high accuracy.

### 3.6. Decision Trees

Decision trees represent decisions in the tree form where leaves are labeled with class attributes and inner nodes represent the attributes in descriptive form. They are most popular in data mining. It is made upside-down with the root as the top node. They make the interpretation quite easy and simple, and this is the main reason behind there usage. For a given node *X*, the children of *X* corresponds to all the values that could be possible of associated attributes. They are robust to noisy data. The algorithm starts with choosing the best characteristic which produces most information for the categorization process. Process will end when all the leaf nodes become pure (all instances belong to the same class) or when no additional classification is required [63].

### 3.7. Random Forest (RF)

RF proposed by Leo Breiman and Adèle Cutler in 2001 is a well-known machine learning classifier. It is an ensemble method that works by combining the concepts of subspaces and “bagging” [64]. RF builds a set of decision trees from the available training dataset [65]. The label is decided after collecting votes from several decision trees. It is one of the best classification algorithms for accurately classifying large datasets. The applications of RF include drug discovery, remote sensing, network intrusion detection, and remote sensing.

### 3.8. Multilayer Perceptron

MLP is sub part from feed-forward artificial neural networks (ANN). ANN reflects the phenomena in which brains of all humans work. The way the brain receives input, comprehends it, and generates responses is the main inspiration behind ANN. ANN can learn through input data and relate it with the output variable that is desired. Perceptron is the basic unit of artificial neural networks. Each perceptron takes some weighted input and generates output using some activation function. They have multiple existing applications as character recognition, data compression, pattern recognition, computer vision, speech recognition, and protein secondary structure.

### 3.9. Convolutional Neural Network (CNN)

Increased number of parameters in MLP and its complicated architecture made it complex to use. Deep learning was introduced to reduce these increasing numbers of parameters. The most popular class of deep learning is CNN. Since the past decade, it has been used in various fields such as pattern recognition and image processing. The abstract features are obtained as the input propagates towards deep layers. The main advantage is that they use little preprocessing in comparison with other image classification algorithms. The main problem with CNN is it cannot be implemented on temporal data.

### 3.10. Recurrent Neural Network (RNN)

RNN is used to deal with sequential data and recognize the patterns in it. The main idea behind creating RNN was to use it to process temporal data. Just like ANN, RNN has neurons with three distinct layers (input, hidden, and output). The difference from traditional ANN lies in the hidden layers. This layer has a temporal loop that enables RNN not just to produce output but also to feed this output to itself. In this way, they sort of develop short-term memory. They remember the sequence; due to this ability, they have widespread usage in various fields. They have applications in NLP, machine translation, speech recognition, and text summarization.

### 3.11. Long Short-Term Memory (LSTM)

LSTM is a type of artificial recurrent neural network which is used in deep learning techniques. Feed forward neural network does not have feedback connection but LSTM hasthem. It can process both single data point like one image or one word and whole sequence like whole video or whole text. It consists of input gate, forget gate, output gate ,and cell. Cell holds value for each interval while remaining gates control flow of information inside and outside of cell. RNN suffers from disappearing gradient problem during back propagation, as weights are upgraded through gradient. So, LSTM solves this issue by using gates inside structure which regulate the flow inside and outside the cell as mentioned earlier. It is widely used in speech analysis, text generation, and speech recognition.

### 3.12. Gated Recurrent Unit (GRU)

GRU was introduced in 2014 by Kyunghyun Cho. It is like LSTM combined with a forget gate, but it has less constraints than LSTM. We can also describe it as a gated phenomenon in RNN. It has shown its performance better or equal to long short-term memory in many tasks such as speech and music signal models as well as in NLP tasks, but it has been analyzed that it shows good and accurate performance on less datasets. It also eliminates the vanishing issue of gradient problem using update and reset gates phenomena. These gates worked as vectors and decide which part of information should be displayed as output, and these gates can hold the irrelevant information for a long time which is its specialty. If they are trained very well, they can produce highly accurate results on complex datasets. GRU is used by plenty of researchers in many real world problems.

## 4. Methodology

The methodological approach can be summarized in four main steps:

### 4.1. Data Set

Dataset used in this research work is titled as “COVID Fake News Dataset” developed by (Sumit Banik, 2020) and published on *Coronavirus Disease Research Community-Covid-19*. Dataset contains 10202 COVID fake news shared all over social media platforms including Facebook, Instagram posts, and news on social media with the keywords COVID-19, coronavirus, and pandemic. Dataset is organized in two columns. First column title is headlines, and second column title is outcome. First column contains strings attributes, and second one contains binary labels 0 and 1. O indicates headline is fake, and 1 indicates headline is real.

### 4.2. Data Preprocessing

Fake news on COVID-19 must be cleaned during the preprocessing step; during this phase, we apply several cleaning and filtering techniques on these fake news on COVID-19 such as removing links, identifiers, deleting words that contain several less than 3 characters, and filtering empty words.

### 4.3. Data Vectorization

Transformation of texts to digital vectors because most automatic learning algorithms do not take text directly but digital vectors for that performs a transformation of text to digital vectors based on the bag-of-words technique with the TF-IDF method for calculating the score of each word.

### 4.4. Classification Model Building

We choose the most efficient classification algorithm based on the results, and then we built our classification model.

### 4.5. Model Evaluation and Testing

Training and evaluation of classification model by performance measures (confusion matrix, classification rate) test the model on a set of test data that represents a set of unclassified fake news on COVID-19, to predict the sentiment class of each fake news on COVID-19 among this set.  Figure 1 shows the architecture of our classification system.

For evaluation purposes of performance, we have computed five metrics. Precision is percentage of related cases between all the regained occurrences, where recall is basically the division of the sum of relative documents that are regained. We count the average of both recall and precision that is called F1-score. On the other hand, confusion matrix is measurement of different parameters that are used to evaluate the performance of classification algorithms.

According to the results obtained in this study, to analyze the feelings of fake news on COVID-19 using text mining and data mining techniques, we used thirteen different classifiers: random forest, support vector machine, *K*-nearest neighbor, Naïve Bayes, logistic regression, decision tree, Adaboost, MLP, CNN, LSTM, Bi-LSTM, GRU, and RNN. From the comparison of the different measures, we find that BiLSTM and CNN perform better than other learning methods even though machine learning algorithms give a good accuracy, but CNN and BiLSTM are the most efficient because they gave a very high accuracy of 97%. Consequently, we find that CNN and BiLSTM are the most efficient classifiers to build a model for classifying fake news on COVID-19 sentiment. Our automatic learning model can only process numerical values as vectors or matrices. To prepare our fake news on COVID-19 for the automatic learning model, we create a reverse document frequency vectorization (TF-IDF) term. The result of this vectorization is a hollow matrix that contains a representation of each sentence as a vector, and the vector has the same length as our vocabulary, i.e., the list of all the words observed in our learning data, each word representing an entry in the vector.

For the evaluation of the model's performance, we will perform a test on a separate test set, to estimate the performance of the generalized model.

Table 1 shows eight classification models that have been validated using evaluation metrics such as precision, recall, and F1-score, while Table 2 shows these results with corresponding macro and weighted average.

Table 3 shows five deep learning algorithm-based results while Table 4 shows deep learning-based models results according to precision, recall, and F1-score. Results of the experiment have shown that CNN and BiLSTM outperform in all aspects such as execution time, nonsensitive to outliers, and the reduction of noise. The results obtained using the classification algorithm outshines using real samples obtained from the reliable repository. For all the experiments in this section, the performance shown is based on the test dataset.

Figures 2–14 explain how the dataset has been handled by a data analysis technique and visualization tool used to apply color in the bar graph to represent height and width called a heat map. It is very useful in visualizing the concentration of values between two dimensions of a matrix and helps in finding patterns and gives a perspective of depth. Here, we applied a heat map to observe the data. Hence, the generalized view of numeric values for our dataset is obtained. In our case, the heat map is displaying various attributes.

Figures 15 and 16 demonstrate the performance metrics: precision, recall, and F1-score which ranges from 0 to 1. Whenever the system performs well, the value will be 1.

## 5. Comparative Discussion

The findings of all machine learning-based models that were tested can be seen in the aforementioned figures and tables. All of the classifiers performed admirably; although, certain classifiers outperformed others in terms of precision, recall, f1-score, and accuracy, when compared to other machine learning classifiers. We have tested various models on a large dataset comprising COVID-19 false news. We have divided our dataset into two halves, one for training and one for testing, in the following manner: each with an 80 percent and a 20 percentage of false news, respectively. *K*-nearest neighbor, multilayer perceptron, and random forest are the most accurate machine learning classifiers, with 97 percent accuracy. 96 percent accuracy was attained using logistic regression, decision tree, support vector machine, and AdaBoost, while Naive Bayes obtained 95 percent accuracy. When we have analyzed the accuracy, recall, and f1-score, random forest reigns supreme with precision, recall, and f1-score of 0.99, 0.98, and 0.98, respectively. Multilayer perceptron placed second with accuracy, recall, and f1-score of 0.98, 0.98, and 0.98, respectively.

## 6. Comparative Discussion

The findings for deep learning-based classifiers can be found in the tables and figures described earlier. In this research, we employed five deep learning-based classifiers including LSTM, BiLSTM, GRU, RNN, and CNN. We measured their performance using a variety of measurements, such as precision, recall, accuracy, and the F1-score. According to the results, CNN and BiLSTM scored the greatest accuracy of 97 percent among all of these frequently used classifiers. On the other hand, LSTM, GRU, and RNN achieved 95 percent accuracy rate. The results clearly demonstrate that deep learning classifiers are excellent at classifying false news on a particular subject. These classifiers are also the most efficient in terms of time, speed, and processing. For CNN and BiLSTM, the precision, recall, and F1-score increased by 0.97, 0.97, and 0.97, respectively, while LSTM, RNN, and GRU improved their accuracy, recall, and F1-score by 0.91, 0.95, and 0.93, respectively.

## 7. Conclusion

In our research, eight machine-learning algorithms such as Naive Bayesian, Adaboost, *K*-nearest neighbors, random forest, logistic regression, decision tree, neural networks, and support vector machine and four deep learning CNN,LSTM, RNN, and GRU are employed to detect sentiments on fake news on COVID-19. We audited various techniques and conducted experiments on the dataset from a reliable repository to find or adapt the best classifier for the sentiment analysis. Furthermore, the system has been analyzed in the aspects of precision, recall, and F1-score for all the algorithms.

In future, we aim to use a large and complex dataset, and the number of labels can also be increased. We can include other languages also and use special characters and numeric values as well. It would be valuable to include the emoticons as they are widely used in social media to represent the expressions. Also, we will try to use the Twitter streaming API to retrieve tweets in real-time in order to do a real time sentiment analysis and exploring other social networks.

## Figures and Tables

**Figure 1:** Research methodology.

**Figure 2:** Heat map of logistic regression.

**Figure 3:** Heat map of random forest.

**Figure 4:** Heat map of decision tree.

**Figure 5:** Heat map of SVM.

**Figure 6:** Heat map of KNN.

**Figure 7:** Heat map of AdaBoost.

**Figure 8:** Heat map of MLP.

**Figure 9:** Heat map of Naïve Bayes.

**Figure 10:** Heat map for CNN.

**Figure 11:** Heat map for LSTM.

**Figure 12:** Heat map for bi-LSTM.

**Figure 13:** Heat map for GRU.

**Figure 14:** Heat map of RNN.

**Figure 15:** Classification accuracy machine learning-based approaches results for fake news on COVID-19.

**Figure 16:** Classification accuracy deep learning-based approaches results for fake news on COVID-19.

**Table 1:** Machine learning based approaches results for fake news on COVID-19.

Model	Accuracy	Precision	Recall	F1-score
Logistic regression	96	0.99	0.97	0.98
Random forest	97	0.99	0.98	0.98
Decision tree	96	0.96	0.96	0.96
SVM	96	0.99	0.97	0.98
KNN	97	0.97	0.96	0.98
Adaboost	96	0.98	0.97	0.97
MLP/BPA	97	0.98	0.98	0.98
Naïve Bayes	95	0.99	0.97	0.98

**Table 2:** Macro and weighted average of precision, recall, and F1-score.

Metrics	Average	Machine learning classification algorithms							
		Logistic regression	Random forest	Decision tree	SVM	KNN	Adaboost	MLP/BPA	Naïve Bayes
Precision	Macro	0.64	0.73	0.75	0.68	0.51	0.66	0.74	0.69
	Weighted	0.99	0.99	0.96	0.99	1.00	0.98	0.98	0.99

Recall	Macro	0.99	0.99	0.76	0.99	0.98	0.85	0.90	0.97
	Weighted	0.97	0.98	0.96	0.97	0.96	0.97	0.98	0.97

F1 score	Macro	0.71	0.81	0.76	0.76	0.51	0.71	0.80	0.77
	Weighted	0.98	0.98	0.96	0.98	0.98	0.97	0.98	0.98

**Table 3:** Deep learning-based approaches results for fake news on COVID-19.

Model	Accuracy	Precision	Recall	F1-score
LSTM	95	0.90	0.95	0.93
BiLSTM	97	0.97	0.97	0.97
GRU	95	0.91	0.95	0.93
RNN	95	0.91	0.95	0.93
Conv1d	97	0.97	0.97	0.97

**Table 4:** Macro and weighted average of precision, recall, and F1-score of DL.

Metrics	Average	Deep learning classification algorithms				
		CNN	LSTM	Bi-LSTM	GRU	RNN
Precision	Macro	0.64	0.79	0.71	0.85	0.47
	Weighted	0.97	0.90	0.97	0.91	0.91

Recall	Macro	0.98	0.96	0.96	0.67	0.50
	Weighted	0.97	0.95	0.97	0.95	0.95

F1 score	Macro	0.71	0.80	0.80	0.79	0.48
	Weighted	0.97	0.93	0.97	0.93	0.93

## Data Availability

This work is part of the MS thesis of the student. The data is not available until the thesis defense. In case of any queries, do let me know.
